# Perception of Individuals with Diabetes about Efficacy and Safety of Complementary and Alternative Medicines (CAM) in the Jazan Region, Saudi Arabia

**DOI:** 10.1155/2022/2104056

**Published:** 2022-05-05

**Authors:** Abdulkarim M. Meraya, Waquar Ahsan, Mohammed Albratty, Hassan A. Alhazmi, Asim Najmi

**Affiliations:** ^1^Department of Pharmacy Practice, College of Pharmacy, Jazan University, Jazan, P. O Box No. 114, Saudi Arabia; ^2^Department of Pharmaceutical Chemistry and Pharmacognosy, College of Pharmacy, Jazan University, P. O Box No. 114, Jazan, Saudi Arabia; ^3^Substance Abuse and Toxicology Research Centre, Jazan University, P. O Box No. 114, Jazan, Saudi Arabia

## Abstract

**Background:**

CAM is widely accepted for the management of diabetes, and CAM users from many countries showed positive perception towards its use. However, little is known about the perception of individuals with diabetes in Saudi Arabia.

**Objectives:**

This study was aimed to assess the perception of the individuals with diabetes of Jazan region in Saudi Arabia towards CAM.

**Methods:**

An online, anonymous cross-sectional survey was designed and conducted between September 5 and December 31, 2021. Data were collected using 19-item self-report survey from the individuals with diabetes of the Jazan region.

**Results:**

A total of 359 validated responses were received. Approximately, 34% of the participants reported using CAM with modern medicine to control diabetes. Most of the participants reported that CAM is affordable, accessible, acceptable, and effective. Of the study sample, 28% reported using herbal medicine to control diabetes. Significantly, higher percentages of CAM users reported media (42% vs 27%) and friends/family (31% vs 27%) as the primary sources of information about CAM as compared to non-CAM users. Individuals who used CAM for diabetes showed significantly more positive perception (*β* = 2.386; *p*=0.001) than those who did not use CAM in the adjusted analysis. Similarly, students had a significantly higher positive perception towards CAM (*β* = 4.121; *p*=0.013) compared to employed individuals.

**Conclusion:**

A quarter of the sample of individuals with diabetes used herbal medicine to control diabetes. Individuals who ever used CAM for diabetes showed positive perception towards CAM. However, there is a need of healthcare workers to be involved in educating the individuals with diabetes and the general public in order to use CAM more effectively and safely.

## 1. Introduction

The increasing prevalence of type 2 diabetes mellitus (T2DM) has been a cause of concern worldwide as the number of T2DM cases has tripled from 151 to 463 million worldwide from 2000 to 2019 [1]. This number is expected to rise further and, by the year 2045, it is believed to reach 700 million [1, 2]. A staggering 10% (760 billion USD) of the total global health expenditure is spent on the treatment of diabetes, and a whopping 4.2 million deaths are accounted alone for diabetes [3]. The Kingdom of Saudi Arabia had seen an alarming increase in the prevalence rate of DM from 9% in 1980 to 22% in 2008, and a study in 2016 reported an estimated 7 million confirmed patients with diabetes and approximately 3 million being prediabetic [4, 5]. Saudi Arabia is among the top 3 countries in the Middle East and North Africa (MENA) region with highest estimated number (27,800) of children and adolescents (0–19 years) diagnosed with type 1 DM in the year 2019 [1]. Currently, Saudi Arabia is ranked 7^th^ worldwide for having new cases of type 1 DM per year. Lifestyle habits including unhealthy diet and sedentary and inactive lifestyles are one of the most important factors leading to T2DM.

Among many therapies for DM, use of complementary and alternative medicines (CAM) has been a popular choice for a large number of populations. The CAM can be defined as a group of medical and healthcare systems, products, and practices, which are not part of currently used conventional medicines. Usage of CAM as an alternative to the conventional therapy of many diseases is becoming increasingly popular, and it is believed that 80% of the world population uses CAM for primary health care [6]. CAM not only includes the use of herbal medicines, but it also includes acupuncture, hijama, moxibustion, faith healing, massage therapy, music therapy, and hypnosis [7]. The major reasons behind the use of CAM are easy availability, more affordability, strong belief about their efficacy, and lesser-perceived side effects associated with CAM in comparison to the prescription drugs [8].

Previously, several surveys have been conducted to assess the use of CAM in patients diagnosed with diabetes. These studies have reported the use of CAM for the treatment of T2DM by 25–57% of patients and the diabetics are 1.6 times more likely to use CAM in comparison to the nondiabetics [9–11]. In one such study conducted on Canadian population, 502 patients with diabetes responded to the survey and 44% of the respondents reported to have used over-the-counter supplements and 31% took alternative medications for the treatment of diabetes [12]. Similar survey conducted in the United States at national level revealed use of CAM by 57% patients with diabetes in the previous year [13]. An Australian study reported 25% people with diabetes to have used CAM in the previous 5 years [14]. A cross-sectional survey on 326 patients with diabetes from Taiwan showed use of CAM by 22.7% patients before and 61.0% after being diagnosed for diabetes [15]. Nutritional supplements were among the most used CAM both before and after diagnosis. Interestingly, only 24.6% patients using CAM reported to have revealed this to their healthcare professionals [15]. Nevertheless, little is known about the CAM use in the Jazan region and Saudi Arabia in general [16–18].

As the efficacy of CAM in diabetes still lacks good supportive evidence, self-administration with or without conventional medicines can lead to ineffective management of diabetes and unprecedented adverse effects and might result into a delayed or even failed therapy. Estimation of population using CAM for the treatment of diabetes is important to know and the use of CAM should be considered clinically while prescribing the antidiabetic drugs. Since most of the patients use CAM in conjunction with the prescription drugs, not as an alternative medicine, these patients should be educated well about the safe use of CAM and should be encouraged to reveal the use of CAM to their physicians and get their opinion and required adjustments in the therapy. The aim of this study was to assess the perception of individuals with diabetes of the Jazan region about CAM in order to identify its pattern of use, reasons to use, and perception towards its efficacy and safety.

## 2. Materials and Methods

### 2.1. Study Tool

An anonymous online cross-sectional survey was used to collect data for this study which was conducted during September 5 to December 31, 2021. The survey was prepared as a self-report survey using Google forms, and the anonymity of respondents were maintained throughout the survey. The link for the survey was circulated to various hospitals, healthcare centers, and various social media platforms such as Twitter and WhatsApp, among male and female respondents who had diabetes, among those who were above the age of 18 years, and those who were residing in the Jazan region of Saudi Arabia. The convenience sampling method was used for sampling in this study. The perception towards CAM was measured using a 7-item scale. Individuals with diabetes were asked about CAM and indicate their agreement/disagreement on a 5-point scale from strongly disagree to strongly agree for the following statements: (1) CAM is effective in diabetes; (2) CAM is safer than modern medicine; (3) CAM should be integrated with modern medicine; (4) prefer first to visit CAM practitioner than modern medicine; (5) recommend a sick person first to visit CAM practitioner; (6) CAM is more affordable than modern medicine; and (7) CAM has no side effects.

Several quality control measures were employed to ensure that the study was appropriately done. These included the wide publicity of the questionnaire, proper designing of data collection instrument, pilot or pretest survey, and appropriate data collection and processing. Questionnaire was designed and prepared by authors and was reviewed and validated by a six-membered independent expert committee. A pretest or pilot survey was also conducted on 40 participants prior to the main survey in order to assess the ease of use and to determine the time for completion. It also helped to establish the clarity, understandability, and proper sequencing of questions. The collected data were checked for consistency and missed response, if any, and were processed further to obtain the accurate and precise results.

### 2.2. Inclusion and Exclusion Criteria

Any male or female participant who had been diagnosed with diabetes, who were above the age of 18 years, residing in any city or village of the Jazan region, willing to participate in the study, and willing to give the informed consent were included in the study. The participants not fulfilling any of these criteria were excluded from the study.

### 2.3. Study Questionnaire

The survey questionnaire comprised three major sections. The section one comprised six questions asking the sociodemographic status of the participants including age, gender, marital status, education status, employment status, and area of living. The second section of the survey comprised seven questions related to the source of information about CAM, type of diabetes, knowledge of CAM, usage, reasons for using CAM, and discussion of CAM use with physicians were asked. Finally, the third section aimed at assessing the perception of individuals with diabetes on CAM usage consisted of six questions; regarding the efficacy, safety, affordability, associated side effects, preference to visit CAM practitioner, and recommendation of a person with diabetes to CAM practitioner.

### 2.4. Sample Size

The sample size was determined using the procedure described elsewhere [19]. The following formula was used to calculate the sample size:

(1) $$\begin{array}{c} \text{sample size}\left(n\right)=\frac{Z_{1-\alpha /2}^{2}P\left(1-P\right)}{d^{2}}, \end{array}$$

where *Z*_1−*α/2*_ = standard normal variate which was considered to be 1.96 for 5% type 1 error (*p* < 0.05), *P* = expected prevalence of CAM use among patients with diabetes (30%) based on previous literature [20], and *d* = absolute error or precision (0.05). A sample size of 323 patients were obtained from the formula. However, to reduce the chances of error, a sample size of 359 patients was taken using the convenience sampling method.

### 2.5. Informed Consent Form (ICF)

An informed consent was obtained from each participant before the start of the survey. They were informed about the survey, types of questions, criteria for participation, and necessity of the survey and were asked to answer a mandatory question asking about their willingness to participate in the survey in the form of “Agree” or “Do not Agree.” The minimum criteria for age (18 years or above) and location (Jazan province) were provided to the respondents and they needed to agree to the criteria before attempting the survey. Respondents less than 18 years of age or from outside Jazan province were asked to disagree to the ICF and leave the survey. Participants clicking on “Agree” could only proceed further, whereas clicking on “Do not Agree” ended the survey.

### 2.6. Ethical Considerations

The study protocol, informed consent form, and the survey questionnaire were submitted to the Institutional Research Review and Ethics Committee of Jazan University and prior approval were taken (Approval no. REC42/1/145).

### 2.7. Statistical Analysis

The statistical analysis was performed using the STATA 16. For the categorical variables, frequency and percentages were calculated. Means and standard deviations were computed for continuous variables. To determine the associations between sociodemographic factors and CAM use status, the chi-square test or Fisher's exact test was employed. Internal reliability for the perception scale was tested using Cronbach's alpha. Exploratory factor analysis using principal component analysis extraction was performed for perception scale. The Kaiser–Meyer–Olkin measure of sampling adequacy and Bartlett's test of sphericity were used to determine the suitability of the data for factor analysis [21]. In addition, Velicer's minimum average partial test was conducted to determine the number of factors [22]. Unadjusted and adjusted ordinary least-squares regression with heteroskedasticity-robust standard errors option was conducted to examine the relationships between the explanatory variables and perception toward CAM. Variables with *p* values < 0.05 were considered as statistically significant.

## 3. Results

The present survey was aimed to assess the perception of CAM usage, efficacy, and safety among individuals with diabetes present in the Jazan region of Saudi Arabia. A total of 493 participants attempted the survey, out of which 40 were not from Jazan and 80 did not have diabetes. Furthermore, 14 were excluded because of missing information on CAM use. Therefore, the total number of accepted and validated responses was 359. The mean age of the participants was 46.3 (SD = 15.2).  Table 1 shows descriptive statistics of the participants. A majority (53.4%) of the participants had type 2 diabetes, 29.3% had type 1, whereas 17.3% respondents did not know the type of diabetes they have. More than half of the respondents (59.6%) have heard of CAM; however, 39% of respondents did not hear about CAM before. When asked about the use of CAM, the majority of respondents (66.3%) reported that they did not use CAM together with modern medicines for the treatment of diabetes, while 33.7% used CAM in combination with the modern medicines. Almost three-quarters (73.5%) of respondents did not reportedly use the CAM in the past two years. More than one-quarter (28%) of the respondents reported using herbal medicine for diabetes. When the respondents were asked about the reason(s) of using CAM for the treatment of diabetes, affordability, accessibility, acceptability, and effectiveness all were selected by majority (54.6%) of the participants, followed by accessibility alone (17.8%) and acceptability alone (14.5%). Interestingly, most of the respondents (67.4%) reported that they never discussed the CAM practice with their physicians, and 25.6% discussed it sometimes. Merely 7% of the participants who used CAM discussed its use with the physicians.

The sociodemographic characteristics by CAM use of all respondents are summarized in Table 2. These variables were compared among the CAM users and CAM nonusers. The gender distribution among the study samples was found to be almost equal as among the CAM users: male participants were 51.2%, whereas females were 48.8%. Similar distribution was seen among the CAM nonusers as percentage of male (50.4%) and female (49.6%) respondents was almost equal. Majority of the participants were married as 71.9% among the CAM users and 66.8% among the CAM nonusers were reported to be married. Similarly, when the educational status of respondents was asked, almost half reported to have education more than high school among both CAM users (49.6%) and CAM nonusers (51.7%). Furthermore, more than half of the respondents were employed among both CAM users group (61.2%) and CAM nonusers group (57.6%). A similar trend was observed when the respondents were asked about the area of living as more than half of them were from the rural area among CAM users (57%) and CAM nonusers (60.5%). Interestingly, a very important and highly significant (*p* < 0.001) finding of our study was that the majority of participants who were CAM users reported media (42.1%) as their primary source of information about CAM followed by family and friends (30.6%). Also, majority of the CAM nonusers (53%) reported media and friends and family as their major source of information, followed by others (42.9%).

The mean score for perception towards CAM was calculated to be 23.1 (SD = 6.5), and the Cronbach's alpha for the scale was 0.92. The results of exploratory factor analysis indicated that one-factor explained 99.9% of the variance. The Kaiser–Meyer–Olkin measure of sampling adequacy was 0.892 and the Bartlett's test of sphericity gave a *p* value of <0.001, indicating that data are adequate for factor analysis. Velicer's minimum average partial test also indicated one-factor solution.  Table 3 displays unadjusted and adjusted relationships between the explanatory variables and perception towards CAM. In the unadjusted analysis, a significant relationship was found merely between CAM use for diabetes and perception towards CAM. Individuals who used CAM for diabetes had significantly more positive perception (*β* = 2.612; *p* < 0.001) than those who did not use CAM. Similarly, there was a significant relationship between CAM use and perception toward CAM after controlling for age, sex, marital status, education level, job status, and area of living. Individuals who used CAM for diabetes had significantly more positive perception (*β* = 2.386; *p*=0.001) than those who did not use CAM. Furthermore, students had a significantly higher positive perception towards CAM (*β* = 4.121; *p*=0.013) compared to the employed individuals in the adjusted analysis.

## 4. Discussion

Saudi Arabia is one of the countries of the world where the number of new diabetes cases is increasing rampantly, and the government agencies are putting enormous efforts in educating people about the disease emphasizing its prevention and treatment [5]. Saudi Arabia is one of the countries which holds strong cultural and traditional values, and the use of CAM as a folklore for the treatment of many diseases is a part of their tradition since many years [23]. Saudi Arabia is blessed with plethora of medicinal herbs in almost every part of the country, which have been used by many herbalists and CAM practitioners since hundreds of years. The knowledge about use of CAM for the treatment and management of ailments is being passed from one generation to other and is widely accepted irrespective of the area of living. People living in the cities also have similar beliefs and acceptability for CAM as the ones living in villages have [24, 25]. Even the educational status does not change the perception of CAM users.

This study was aimed to assess the usage pattern, reasons for use, and the perception about the safety and efficacy of CAM among individuals with diabetes of Jazan region, Saudi Arabia. The opinion of CAM users and CAM nonusers were obtained, and the association of CAM usage with sociodemographic factors of the respondents was also measured. Importantly, the sociodemographic factors such as age, gender, marital status, educational status, and area of living did not influence the CAM usage among the respondents as no significant association was observed between them showing their strong belief about the efficacy of CAM. These results were consistent with the previously reported studies on the Saudi Arabian population [20, 26] as well as non-Saudi population [27], where no significant association was observed between the demographic variables and the use of CAM.

In this study, it was observed that among both the CAM users and CAM nonusers, the primary source of information through which they get information about CAM is either media or their family and friends. More than 70% of the CAM users and more than 50% of CAM nonusers relied on these two sources for the information they needed about CAM. This shows that there exists a lack of proper understanding among the respondents about the reliable and authentic sources for CAM-related information. Also, the information present on the authentic platforms should be widely publicized and this needs urgent government intervention. Keeping in view the large population living in rural areas and in the interior parts of the country; proper, authentic and reliable information about CAM usage, efficacy, and safety should be disseminated to general public using appropriate means. Sometimes, the efficacy of any herbal drug is overstated and is rumored without any proper evidence which could lead to harmful side effects [28, 29].

In the second part of the survey, when the respondents were asked about the use of CAM together with modern medicines for the treatment of diabetes, 33.7% patients responded that they used both therapies in conjunction and more than two-thirds (67.4%) never discussed the use of CAM with their physicians. This again calls for an awareness drive among the CAM users as the use of CAM together with modern medicines is still not established owing to the lack of strong evidence in most of the cases. The use of CAM might potentiate or counter the allopathic therapy using modern medicines and can even lead to delay or failure of the therapy [30–32]. It is always advisable to discuss the CAM use with the physicians as they can make proper adjustments to the therapy and can suggest appropriate ways to use CAM with the modern medicines.

Affordability, accessibility, acceptability, and effectiveness all together were reported by most of the respondents as their reasons to use CAM as it is easily available and accessible in most of regions of Saudi Arabia, especially the remote ones. Also, CAM is already tried and tested by their acquaintances who give positive feedbacks on its use testifying its efficacy. Common people have a general perception that CAM either does not cost money or are relatively much affordable than the modern medicines and this is also one of the reasons for its use [33]. A similar perception exists for the side effects of allopathic medicines, as most of the people believe that modern medicines have serious side effects especially if they are being used for a prolonged period. CAM, on the other hand, either does not have these side effects or are relatively much safer to use.

These perceptions of respondents were further assessed in the third part of the study where the questions regarding the effectiveness, safety, affordability, visit to a CAM practitioner, and recommendation to a CAM practitioner were asked. The average score of the perception scale was 23.1, indicating a positive perception towards CAM. Although CAM includes therapy by other means too, the use of herbal drugs or naturopathy is the most common form of CAM [34]. This widespread acceptability and usage of CAM might signify the dissatisfaction with the allopathic system of medicine owing to its perceived side effects. The possibility of drug-herb interaction is ignored while taking modern medicines together with the herbal drugs.

Naturopathy might include the use of herbs, plant extracts, fruits, vegetables, or minerals, and in most of the cases, their synergistic action with different antidiabetic drugs are still unknown or less-studied [13]. The average score of the perception scale in our sample indicated that individuals with diabetes perceive CAM as safer and more affordable than modern medicine. This showed a lack of discernment among the general population about the affordability of CAM in comparison to the modern medicines as few herbal drugs or even traditional therapies cost very high to the patients which easily surpasses the cost of modern medicines [33]. Also, Saudi Arabia has highly developed government healthcare services which are accessible to all its citizens and residents, and all the necessary medicines are freely available in government-run hospital pharmacies. Similarly, a good percentage of CAM users and nonusers also had the perception that CAM does not have any side effects. They should be educated that despite the benefits that CAM and associated therapies might offer, some of the herbal products can be toxic especially if they are not used properly [35]. The improper use of CAM may even worsen the diabetic complications, and the healthcare providers should discuss and educate the patients with evidence-based facts regarding the proper use and safety of CAM along with the potential interactions of CAM interventions with their antidiabetic therapy.

The strength of our study is that individuals with diabetes from all over Jazan province including villages and cities were included. This study would add a new dimension to the literature as this is the first of its kind in this region assessing the CAM use in individuals with diabetes and their perception about its efficacy and safety. This study also has some limitations as being an online cross-sectional study. We included the respondents who could use the Google forms to answer. The sample mostly consisted of well-educated individuals, and therefore, there can be a sampling bias. To address the sampling bias, the questionnaire was distributed using several online channels such as social media apps, emails, text messages, and QR codes in order to improve the visibility among different respondents. The questionnaire was also distributed to various hospitals and healthcare centers of the Jazan region to get maximum patient outreach. This study used the self-report questionnaire; therefore, there can also be recall and response bias which was addressed using anonymous survey and using neutral and nondeceptive questions. Furthermore, this study failed to determine the type of CAM patients with diabetes are using as well as the harmful or beneficial effects experienced by them. Owing to these limitations, this study cannot be generalized for the population of the Jazan region and randomized studies with much larger sample size are nevertheless needed to find the predictors of CAM usage in this region.

## 5. Conclusions

This study can be implicated into an urgent need and call for policy makers of this region to create proper regulatory guidelines and tools for the marketing of CAM products for their safe use. An appropriate awareness drive or campaign should be initiated in order to educate common people about the effectiveness, proper use, safety concerns, herb-drug interactions, herb-herb interactions, possible minor and major side effects of CAM, etc. Many people still depend on the advertisements in newspapers and media channels or ask their family or friends for their queries about CAM, and this could lead to improper use of the CAM therapy. There should be a provision or an authentic source which can be accessible to everyone and can provide all the relevant information and answer the general queries and doubts about the CAM use. The healthcare providers also have a major role to play here as they need to build trustworthy relationships with their patients so that they can share their CAM use freely and discuss the pros and cons of the two therapies if used concomitantly.

## Figures and Tables

**Table 1:** Descriptive statistics of the sample.

Questions	*n* (%)
*Type of diabetes*	
Type 1	105 (29.3)
Type 2	191 (53.4)
I do not know	62 (17.3)

*Have you ever heard of CAM?*	
Yes	214 (59.6)
No	140 (39.0)
Refused to say	5 (1.4)

*Did you use CAM and modern medicine together for diabetes?*	
No	238 (66.3)
Yes	121 (33.7)

*Did you use CAM in past two years?*	
No	264 (73.5)
Yes	95 (26.5)

*Did you use herbal medicine for diabetes ever?*	
No	258 (72.0)
Yes	101 (28.0)

*Reason for using CAM?*	
Affordability	17 (4.7)
Accessibility	64 (17.8)
Acceptability	52 (14.5)
Effectiveness	30 (8.4)
All of the above	196 (54.6)

*Have you ever discussed CAM practice with physicians?*	
Never	242 (67.4)
Usually	25 (7)
Sometimes	92 (25.6)

**Table 2:** The sociodemographic characteristics and the source of information among users and nonusers of CAM.

Variables	CAM users, *n* (%)	CAM nonusers, *n* (%)	Chi-square (*χ*^2^)	*pp* value
*Gender*				
Male	62 (51.2)	120 (50.4)	0.0216	0.883
Female	59 (48.8)	118 (49.6)		

*Marital status*				
Single	34 (28.1)	79 (33.2)	0.9651	0.326
Married	87 (71.9)	159 (66.8)		

*Education status*				
No education	19 (15.7)	48 (20.2)	2.0629	0.356
≤High school	42 (34.7)	67 (28.2)		
>High school	60 (49.6)	123 (51.7)		

*Employment status*				
Employed	74 (61.2)	137 (57.6)	0.6714	0.715
Unemployed	36 (29.8)	81 (34)		
Student	11 (9.1)	20 (8.4)		

*Area of living*				
City	52 (43)	94 (39.5)	0.4025	0.526
Village	69 (57)	144 (60.5)		

*Source of information about CAM*				
Media	51 (42.1)	63 (26.5)	24.114	<0.001
Educational materials	11 (9.1)	10 (4.2)		
Friends and family	37 (30.6)	63 (26.5)		
Others	22 (18.2)	102 (42.9)		

**Table 3:** Parameter estimates of the explanatory variables from ordinary least-squares regression outcome relative to perception toward CAM.

Explanatory variables	Unadjusted			Adjusted		
	*β*	95% confidence interval	*p* value	*β*	95% confidence interval	*p* value
Age	0.0379	(−0.007–0.083)	0.100	0.05	(−0.007–0.107)	0.087

*Sex*						
Male	*Reference*					
Female	−0.599	(−1.949–0.751)	0.383	0.391	(−1.277–2.059)	0.645

*Marital status*						
Single	*Reference*					
Married	1.119	(−0.399–2.639)	0.148	1.673	(−0.12–3.466)	0.067

*Education level*						
No education	*Reference*					
≤High school	−0.408	(−2.277–1.462)	0.668	−0.537	(−2.612–1.537)	0.611
>High school	−1.181	(−2.893–0.529)	0.175	−1.747	(−3.925–0.43)	0.115

*Job status*						
Employed	Reference					
Unemployed	−0.888	(−2.313–0.5367)	0.221	−1.45	(−3.189–0.29)	0.102
Student	1.486	(−1.018–3.990)	0.244	4.121	(0.883–7.359)	0.013

*Area of living*						
City	*Reference*					
Village	−0.868	(−2.239–0.504)	0.214	−1.168	(−2.554–0.217)	0.098

*CAM use*						
No	*Reference*					
Yes	2.612	(1.241–3.982)	<0.001	2.386	(0.992–3.78)	0.001

## Data Availability

The data used to support the findings of this study are available from the corresponding author upon request.
